The article "Focus on the Analysis of the Effect of Solving the Nursing Mode on the Time of the Production Time of the First Maternity and the Subjective Happiness of the Postpartum" was retracted in 2023. Reasons: signs of a paper mill; suspected computer-generated content; unreliable results or conclusions; lack of ethics approval or compliance.

# Focus on the Analysis of the Effect of Solving the Nursing Mode on the Time of the Production Time of the First Maternity and the Subjective Happiness of the Postpartum

**DOI:** 10.1155/2022/2952949

**Published:** 2022-06-25

**Authors:** Tianmin Zhang, Lingyun Zhang

**Affiliations:** ^1^Characteristic Outpatient Department, Henan Provincial People's Hospital, Zhengzhou 450003, Zhengzhou, China; ^2^Obstetrics and Gynaecology, Henan Provincial People's Hospital, Zhengzhou 450003, Zhengzhou, China

## Abstract

**Objective:**

Focusing to solve the significance of the nursing mode for preliminary maternity care.

**Methods:**

Selected 116 first mothers produced in our hospital from January 2010 to January 2022, which were divided into the control group and research group. The two groups each paid conventional care and focused on solving the nursing mode care. Analyze the two groups of pregnancy endings, self-efficacy, negative emotions, subjective happiness, and analgesics.

**Results:**

The vaginal delivery rate of the research group was higher than that of the control group, and the cesarean section rate, hospitalization time, and delivery process were lower than the control group (*P* < 0.05); the amount of bleeding in the postpartum groups increased, but compared with the control group, the increase in bleeding in the research group was smaller (*P* < 0.05); the research group objective, subjective support, self-evaluation, and subjective happiness index were higher than the control group (*P* < 0.05).

**Conclusion:**

Focusing to solve the nursing model can help the maternal tension relief, the maternal can quickly enter the role, and it plays an important role in establishing a good nursing relationship.

## 1. Introduction

Childbirth is a physiological process for most women, which will cause major damage to the mother, and the maternal is accompanied by obvious childbirth pain [1]. In addition, the strange population and ward environment will cause negative emotions for the first mother, causing changes in their behavior and psychological characteristics. If there is no timely intervention, it will lead to disorders of endocrinology and central nervous system. What is more, postpartum depression occurs [2]. Therefore, in order to improve the end of the pregnancy and improve the sense of happiness of the first maternal and gangsters, the first maternal intervention needs to be provided [3]. At present, there are often two types of analgesia through nondrug and drugs. Nondrug analgesic mainly refers to prenatal guidance and training. Drug analgesic mainly refers to analgesic drugs and anesthesia [4]. In the past, nondrug analgesics were performed in regular care, but due to the lack of targeted and comprehensiveness in the nursing plan, it would interfere with the smooth progress of the plan [5].

The article "Focus on the Analysis of the Effect of Solving the Nursing Mode on the Time of the Production Time of the First Maternity and the Subjective Happiness of the Postpartum" was retracted in 2023. Reasons: signs of a paper mill; suspected computer-generated content; unreliable results or conclusions; lack of ethics approval or compliance.

More and more scholars have pointed out that the focus of focusing on the treatment model can be used in the clinical care of the first mother. This nursing mode was first proposed in the late 1970s. It is mainly used for psychotherapy and consultation. It is an important psychological intervention. Methods have been widely recognized internationally [6, 7]. In order to analyze the feasibility of focusing on the application of nursing models, the nursing method is currently exploring the recovery of the maternal life and the improvement of the psychological state of the mother. I hope to make up for the conventional nursing defects and provide more effective nursing methods for the first mother.

## 2. Data and Methods

### 2.1. General Information

Selected 116 first women produced in our hospital from January 2010 to January 2022. The control group: aged 20–43 years, average gestational week (38.16 ± 2.59) week, average age (25.41 ± 2.37), average fetal double top diameter (9.12 ± 0.45) cm, the average export front and rear diameter (11.36 ± 2.15) CM, and the average diameter (9.53 ± 1.52) cm; the research group: the average gestational week (38.18 ± 2.57) week, aged 20–43 years, the average age (25.42 ± 2.35), the average fetal double diameter (9.15 ± 0.44)) cm, the average export diameter (11.37 ± 2.14) cm, and the average sciatic spine diameter (9.52 ± 1.53) cm. This study has been approved by the ethics department. Different data differences in the two groups are not statistically significant and can be compared (*P* > 0.05).

### 2.2. Methods

#### 2.2.1. Conventional Nursing

For maternal intervention such as health mission, 30 days before and after the expected expenses, obstetric experts conduct analgesic, diet, and psychological guidance for childbirth, once a week, each intervention time is controlled at about half an hour.

#### 2.2.2. Focus on Solving Nursing Mode Care

(1) Understand maternal information: collect information on the medical examination information during pregnancy, understand the status quo of the fetus and maternal and need to establish a good relationship between patients and nursing staff, encourage the maternal behavior to act correctly and need to point out the maternal error behavior in time, and to correct them in time to continuously improve the self-confidence of the maternal. (2) Formation of phased goals: as a nursing staff, it is necessary to explore the problems that occur with the present, formulate solutions, and establish nursing goals. Maternals should also participate in the entire process. By analyzing and solving problems, the joy of success can be experienced, which is conducive to the resolution of subsequent pregnancy problems and the improvement of maternal self-confidence. (3) Explore the goal method: on the basis of the current goals, analysis is the main factors that affect the targets that affect the goals.

The article "Focus on the Analysis of the Effect of Solving the Nursing Mode on the Time of the Production Time of the First Maternity and the Subjective Happiness of the Postpartum" was retracted in 2023. Reasons: signs of a paper mill; suspected computer-generated content; unreliable results or conclusions; lack of ethics approval or compliance.

### 2.3. Observation Indicators

#### 2.3.1. Pregnancy Ending

Record the hospital hospitalization and output time, plots assisted, number of cesarean sections, calculation proportion, and statistics vaginal delivery.

#### 2.3.2. Self-Protection Ability Score

Including four contents of self-responsibility, health knowledge, nursing skills, and self-concepts, the total score is 100 points. The score is proportional to the self-protection ability.

#### 2.3.3. Bleeding Volume

Applying pads to the weight method [8], statistical maternal bleeding amount, bleeding amount = (postpartum hematopoietic pad weight − net weight of care pad)/1.05.

#### 2.3.4. SDS and SAS Scores

By the application of depression self-evaluation table (SDS) and anxiety self-evaluation table (SAS) [9] evaluation of patient depression and anxiety, 53–62 points represent mild depression, anxiety, 63–72 points represent moderate depression, anxiety, and >72 points represent severe depression, anxiety.

#### 2.3.5. Subjective Happiness

By the application of the subjective happiness evaluation table [10] (level 4 scoring method), evaluate objective support, subjective support, self-evaluation, and subjective happiness index.

#### 2.3.6. Satisfaction

By the application of the hospital customized satisfaction metering table [11], evaluate maternal satisfaction: <57 points represent the Disrog cause, 57–75 points represent the satisfaction, and 76–95 points represent very satisfied.

#### 2.3.7. Analing Effect [12]

Level 0 represents painless, level 1 represents mild pain, and level 2 represents need to give drug analgesia, accompanied by obvious pain when performing activity and lying. It is necessary to give strong analgesic drugs and affect normal sleep.

### 2.4. Statistical Method

Data Application Statistics SPSS 22.0 Software was used. If the data meet the normal distribution, (the average ± standard deviation) represents the measurement data, the composition ratio, and the rate description of the counting data. 0.05 explains that there are obvious differences in statistical results. In this study, GraphPad Prism8 software is selected as a figure.

## 3. Result

### 3.1. Two Groups of Pregnancy Ending Comparison

The vaginal delivery rate of the research group is higher than that of the control group, and the cesarean section rate, hospitalization time, and delivery process are lower than the control group (*P* < 0.05) (Table 1).

The article "Focus on the Analysis of the Effect of Solving the Nursing Mode on the Time of the Production Time of the First Maternity and the Subjective Happiness of the Postpartum" was retracted in 2023. Reasons: signs of a paper mill; suspected computer-generated content; unreliable results or conclusions; lack of ethics approval or compliance.

### 3.2. Comparison of the Two Groups of Self-Protection Capabilities Scores

The research group's self-responsibility, health knowledge level, nursing skills, and self-concept scores were higher than the control group (*P* < 0.05) (Table 2).

### 3.3. Comparison of Bleeding Volume of Two Groups

The amount of bleeding in the postpartum group was increasing, but compared with the control group, the increase in bleeding in the research group was smaller (*P* < 0.05) (Table 3, Figure 1).

### 3.4. Two Groups of SDS and SAS Comparison

After nursing, the two groups of SDS and SAS scores were reduced, but compared with the control group, the SDS and SAS of the research group were larger (*P* < 0.05) (Figure 2).

### 3.5. Two Groups of Subjective Happiness Comparison

After nursing, the research group objective, subjective support, self-evaluation, and subjective happiness index were higher than the control group (*P* < 0.05) (Figure 3).

### 3.6. Comparison of Satisfaction of the Two Groups

The control group and research group satisfaction was 77.59% and 98.28%, respectively. The research group satisfied than the control group (*P* < 0.05) (Figure 4).

### 3.7. Comparison of Analgesic Effects in the Two Groups

The analgesic rates of level 0, level 1, level 2, and level 3 of the control group are 3.45%, 32.76%, 46.55%, and 17.24%, respectively. 72.41%, 3.45%, 0.00%. The analgesic effect of the research group is better than the control group (*P* < 0.05) (Figure 5).

## 4. Discussion

The first maternal has no experience in childbirth and insufficient understanding of childbirth knowledge. Therefore, the first mother has a worse degree of psychological tolerance than the maternal psychological tolerance. It is more sensitive to pain and is prone to resistance and fear. This is not conducive to normal delivery [13]. Therefore, according to the characteristics of the primary maternal, the childbirth technical guidance and psychological health education need to be carried out, and the maximum is likely to avoid the impact of risk factors on the end of pregnancy [14]. Focusing on solving, the nursing mode mainly includes 5 aspects of content. Based on the concept of “people-oriented,” considering the characteristics of strength and problems coexisting, constantly cultivate their own resources, improve their potential, pay attention to the advantages of maternal women, and continue to encourage and enlighten them through continuous encouragement and enlightenment. First maternal, let them establish good ideas [15]. In addition, considering the importance of primary maternal and emotional and recovery, help them adapt to the new environment and speed up rehabilitation. Second, the active response emphasizes, not just accepting passive reactions [16].

The article "Focus on the Analysis of the Effect of Solving the Nursing Mode on the Time of the Production Time of the First Maternity and the Subjective Happiness of the Postpartum" was retracted in 2023. Reasons: signs of a paper mill; suspected computer-generated content; unreliable results or conclusions; lack of ethics approval or compliance.

The application of this study focuses on solving the nursing model to care for the first mother. The basis of this care method is psychological theory. It gives individuals full respect and discovers the mother's own advantages and ability. It has been well received by patients and is currently widely used in clinical care for primary women [17]. After the first maternal care for this study, the patient's prenatal and postpartum depression status was significantly adjusted. The main reason is that by collecting the personal data of the first mother, the nursing staff can solve the bad emotional potential of their predecessors. It can take the initiative to participate in the entire nursing plan, which is conducive to solving nursing problems such as prenatal syndrome [18]. Focusing on solution to the nursing mode has been widely used in nursing teaching, health education, and psychological care, especially in improving psychological state [19]. After the first maternal psychological problem is solved, a correct mentality can face childbirth pain, which can alleviate the stress response due to pain. The results of this study show that the analgesic effect of the research group is better than the control group, and the two groups of SDS and SAS scores after nursing are reduced. The results of this study are consistent with the results of the party Yongni and Liu [20]. The results confirmed that compared with conventional intervention methods, the effect of focusing on solving the nursing mode is more obvious. The main reason is that the care method can formulate targeted goals based on the psychological characteristics of the first mother and cooperate with investigation, feedback, and target evaluation. This can be able to a series of problems that occur in the nursing process in efficient and timely resolution [21, 22].

Conventional nursing methods pay attention to the irrigation and teaching of knowledge, but usually do not explore the cause of the problem, which will cause the first mother to have self-guilty psychology. If the status quo is not improved in time, it will be more serious. Application focuses on solving the analysis, answers, and evaluation of the nursing mode to achieve problems [23, 24]. After the preliminary maternal menstruation focuses on solving the nursing mode, the amount of bleeding is significantly reduced, and the hospitalization time and delivery process are shortened. Most of the mothers choose vaginal delivery methods, which is of great significance for maternal and infant health [25]. The good emotions of the first maternal will help the initial women's consumability to increase the consulted by the doctor, and can better accept the arrangement of doctors. Domestic scholars point out that the psychological state of the first maternal is closely related to the subjective happiness, and the subjective happiness is a concept of overall and subjectiveness. It can recognize the quality of life and emotional evaluation [26]. The results of this study show that after nursing, the subjective happiness of the research group is better than the control group. The nursing model gives the first maternal respect and attention and can expect the completion of the next goal. However, we still need to continue to work hard to better improve the focusing mode, expand the application scope of the nursing mode, and continuously practice and explore, further improving the model [27, 28].

The article "Focus on the Analysis of the Effect of Solving the Nursing Mode on the Time of the Production Time of the First Maternity and the Subjective Happiness of the Postpartum" was retracted in 2023. Reasons: signs of a paper mill; suspected computer-generated content; unreliable results or conclusions; lack of ethics approval or compliance.

In summary, focusing on the solution of the nursing model can help the maternal tension relief, the maternal can quickly enter the role, and it plays an important role in establishing a good nursing relationship. The decreased degree of pain after nursing delivery can improve the end of pregnancy, shorten the hospitalization and delivery time, and then improve the mother's self-protection ability and subjective happiness.

## Figures and Tables

**Figure 1:** Comparison of bleeding volume of two groups.

**Figure 2:** Comparison of SDS and SAS of two groups. Compared with the control group, ^*∗*^*p* < 0.05; compared with the intervention of this group, ^#^*p* < 0.05.

**Figure 3:** Two groups of subjective happiness comparison.

**Figure 4:** Both groups' satisfaction comparison.

**Figure 5:** Comparison of analgesic effects in the two groups.

**Table 1:** Two groups of pregnancy ending comparison.

Group	Example	Vaginal delivery	Migrants	Cesarean section	Resident time (*D*)	Past time (min)
Control group	58	27 (46.55)	3 (5.17)	28 (48.28)	3.85 ± 0.74	584.63 ± 48.15
Research group	58	45 (77.59)	4 (6.90)	9 (15.52)	2.35 ± 0.41	462.48 ± 32.84
*X* ^2^/*t*	—	11.864	0.152	14.326	13.503	11.257
*P*	—	<0.001	0.697	<0.001	<0.001	<0.001

**Table 2:** Two groups of self-protection ability score comparison.

Group	Example	Self-responsibility			Health knowledge level			Nursing skills			Self-concept		
		Before care	7*D* after care	14*D* after care	Before care	7*D* after care	14*D* after care	Before care	7*D* after care	14*D* after care	Before care	7*D* after care	14*D* after care
Control group	58	12.18 ± 2.18	15.32 ± 2.21	18.44 ± 2.31	32.78 ± 2.57	37.56 ± 2.89	42.91 ± 3.18	17.13 ± 1.89	21.59 ± 2.07	25.35 ± 2.29	11.07 ± 1.95	13.38 ± 2.16	16.44 ± 2.41
Research group	58	12.86 ± 2.19	20.56 ± 2.56	25.84 ± 2.78	33.19 ± 2.61	42.19 ± 3.16	49.93 ± 3.69	17.43 ± 2.06	28.79 ± 2.17	32.71 ± 2.38	11.68 ± 1.98	18.67 ± 2.57	21.01 ± 2.89
*t*	—	1.676	11.800	15.592	0.853	8.234	10.975	1.676	11.800	15.592	0.853	8.234	10.975
*P*	—	0.097	<0.001	<0.001	0.396	<0.001	<0.001	0.097	<0.001	<0.001	0.396	<0.001	<0.001

The article "Focus on the Analysis of the Effect of Solving the Nursing Mode on the Time of the Production Time of the First Maternity and the Subjective Happiness of the Postpartum" was retracted in 2023. Reasons: signs of a paper mill; suspected computer-generated content; unreliable results or conclusions; lack of ethics approval or compliance.

**Table 3:** Two groups of bleeding volume comparison $\left(\bar{x}\pm s\right)$.

Group	Example	1 h bleeding after delivery	3 h bleeding after delivery	6 h bleeding after delivery	12 h bleeding after delivery	After childbirth, 24 h bleeding volume
Control group	58	142.52 ± 12.42	154.37 ± 15.13	167.24 ± 17.53	181.26 ± 21.16	193.52 ± 24.25
Research group	58	100.31 ± 11.54	112.14 ± 13.58	133.56 ± 16.53	150.38 ± 20.17	164.78 ± 23.49
*t*	—	18.961	15.819	10.646	8.045	6.483
*P*	—	<0.001	<0.001	<0.001	<0.001	<0.001

## Data Availability

The data used to support the findings of this study are available from the corresponding author upon request.
